# The Clinical Value of High-Quality Nursing in Concurrent Radiotherapy and Chemotherapy after Glioma Surgery and Its Influence on the Stress Indicators Cor, ACTH, and CRP

**DOI:** 10.1155/2022/8335400

**Published:** 2022-01-25

**Authors:** Huali Fang, Shanshan Hu, Shanshan Liang, Guangyan Yao

**Affiliations:** ^1^Department of Clinical Laboratory, Yantaishan Hospital, Yantai 264000, Shandong, China; ^2^Department of Neurology (I), Affiliated Qingdao Central Hospital, Qingdao University, Qingdao 266042, Shandong, China; ^3^Department of Neurology, Jinan Central Hospital, Jinan 250013, Shandong, China

## Abstract

**Objective:**

The purpose of this study is to explore the clinical value of high-quality nursing in concurrent radiotherapy and chemotherapy after glioma surgery and its influence on the stress indicators such as cortisol (Cor), adrenocorticotrophic hormone (ACTH), and C-reactive protein (CRP).

**Methods:**

A total of 94 glioma patients diagnosed and treated in our hospital were randomly divided into a research group and a control group, with 47 cases in each group. Both groups of patients were given concurrent radiotherapy and chemotherapy. On this basis, patients in the control group were given basic care, while patients in the research group were given a combination of basic care and high-quality care. The nursing satisfaction and adverse reactions of the two groups were compared. The pain degree and the levels of stress indicators Cor, ACTH, and CRP at different time points were compared between the two groups. The sleep quality, bad mood, and quality of life before and after nursing were compared between the two groups.

**Results:**

After nursing, the nursing satisfaction of the research group (95.74%) was higher than that of the control group (80.85%), and the difference between the two groups was statistically significant (*X*^2^ = 11.678, *P* < 0.05). There was no significant difference between patients in the Visual Analogue Scale (VAS) score and the levels of stress indicators Cor, ACTH, and CRP at the T1 time point between the two groups (*P* > 0.05). With the passage of time, the levels of Cor and ACTH of the two groups showed an upward trend. At T4, the increased levels of Cor and ACTH in the research group were less than those in the control group, and the difference was statistically significant (*P* < 0.05). The VAS scores and CRP levels of the two groups showed an upward trend at T1 and T2 and a downward trend at T3 and T4. And, at T4, the decrease in CRP level of the research group was greater than that in the control group, and the difference was statistically significant (*P* < 0.05). Before nursing, there was no statistically significant difference between two groups of patients in the time to fall asleep, sleep time, number of awakenings, SAS score, self-rating depression scale (SDS) score, quality of life index scores, and total scores (*P* > 0.05). After nursing, the time to fall asleep and the number of awakenings in the two groups of patients showed an upward trend, and the increase in the control group was higher (*P* < 0.05). The sleep time of the two groups showed a downward trend, and the degree of decline in the control group was higher (*P* < 0.05). After nursing, the SAS score and SDS score of the two groups of patients decreased (^*∗*^*P* < 0.05), and the decrease in the research group was more obvious (^#^*P* < 0.05). After nursing, the scores of all indicators of the quality of life and the total score of the two groups increased and the score of the research group increased more significantly (*P* < 0.05). After nursing, the control group had 5 cases of gastrointestinal reactions, 7 cases of bone marrow suppression, 6 cases of leukopenia, 6 cases of thrombocytopenia, and 10 cases of dizziness and nausea. In the research group, there were 1 case of gastrointestinal reaction, 2 cases of bone marrow suppression, 1 case of leukopenia, 1 case of thrombocytopenia, and 2 cases of dizziness and nausea. The difference between the two groups was statistically significant (*P* < 0.05).

**Conclusion:**

Glioma patients are given high-quality care during the course of concurrent radiotherapy and chemotherapy, which can reduce the pain and bad mood of the patient, reduce the stress response of the patient, and improve the quality of sleep and the quality of life of the patient, thereby improving nursing satisfaction and patients compliance, reducing adverse reactions, and having a good prognosis.

## 1. Introduction

Glioma is a common malignant tumor of the nervous system, accounting for about 50% of intracranial tumors. Glioma develops rapidly, with a high mortality and disability rate [1]. The occurrence of glioma is related to environmental carcinogenic factors and congenital high-risk factors [2]. At present, the main clinical treatment for glioma is to surgically remove the tumor tissue, remove most of the tumor cells, relieve the pressure on the peripheral nerve tissue, and improve the patient's quality of life. However, patients often lack the knowledge and understanding of surgical treatment, causing emotions such as fear, tension, and anxiety, and surgery can easily damage the patient's limb function and relapse after surgery. Meanwhile, postoperative radiotherapy and chemotherapy are required, which will produce more adverse reactions, and even some patients will develop drug resistance, which puts patients under greater physical and mental pressure and affects their prognostic recovery [3, 4]. Therefore, it is particularly important to actively carry out nursing interventions for postoperative patients. This study explores the application effect of high-quality nursing care in patients with concurrent radiotherapy and chemotherapy after glioma surgery and aims to provide a reference for the clinical treatment and nursing of glioma. The report is as follows.

## 2. Materials and Methods

### 2.1. General Information

A total of 94 glioma patients admitted to our hospital from May 2016 to January 2019 were selected as the research objects. Each patient was confirmed by pathology and randomly divided into a control group and a research group, with 47 cases in each group. Both groups were given concurrent radiotherapy and chemotherapy after operation. On this basis, the control group took basic nursing, and the research group took basic nursing combined with high-quality nursing. The age of the research group was 25–63 years old, with an average of 47.60 ± 5.37 years old. The age of the control group was 24–60 years old, with an average of 45.90 ± 5.63 years old. There was no significant difference between the two groups of patients in terms of gender, age, BMI, education level, and tumor location (*P* > 0.05) (Table 1). All the specimens of this study were got informed consent from patients. This study was approved by the ethics committee of our hospital.

### 2.2. Selection Criteria

  Inclusion criteria: patients who meet the diagnostic criteria for glioma [5], patients undergoing surgery and receiving radiotherapy or chemotherapy treatment after surgery, patients who voluntarily participate in the study and sign informed consent, patients who have no hearing and language impairment and can communicate normally, and patients with complete clinical data were included.
  Exclusion criteria: patients with other malignant tumors and severe liver and kidney insufficiency, patients with other intracranial diseases, patients with mental disorders, and women during pregnancy or lactation were excluded.

### 2.3. Nursing Methods

Patients in the control group were given routine basic care, including providing patients with a good living environment, keeping the ward clean, maintaining proper temperature and humidity, cultivating a good lifestyle for patients, reducing visiting time and number of people, and avoiding cross-infection. Before the operation, the nursing staff will visit the patient to inform the operation time, operation method and preparations, and other basic information. Routine nursing measures such as vital signs monitoring for patients during surgery are carried out. After the operation, measures such as health promotion and education, routine medication guidance, condition observation, family social support, psychological counseling, and rehabilitation exercises are carried out.

The research group was given routine basic nursing combined with high-quality nursing intervention. The specific method is as follows. After admission, first introduce the patient's room and surrounding environment in detail, so that the patient is familiar with it as soon as possible to eliminate tension. Then, understand its basic situation, according to its specific disease progression; describe in detail the related disease knowledge, treatment plan, and prognosis of intracranial tumors. Emphasize the aspects that require patient cooperation and the importance of active cooperation, and answer patient questions patiently and accurately. The patient should be informed of the operation time and preoperative preparations, fasting, and drinking before 20 : 00 the day before the operation. Provide a quiet and comfortable sleeping environment, requiring patients to rest before 22 : 00. Before entering the operating room, inform the operation procedures and the anesthesia process in detail. Encourage patients, let them relax, and dispel their worries. Real-time monitoring of patient vital signs during the operation was carried out. After the operation, the medical staff should inform the patient of the relevant knowledge of glioma surgery in detail, including precautions, prognosis, radiotherapy and chemotherapy treatment methods, nursing procedures, and their necessity. And strengthen communication and exchanges with patients, and encourage patients to express their inner thoughts. For patients who are anxious, worried, and afraid of bad emotions, nursing staff should provide targeted guidance based on the causes of bad emotions. Carry out daily simple nursing training for patients' family members and accompanying staff, and give positive affirmation to patients' progress. And to give patients as much company and care as possible, become the patient's spiritual sustenance, increase the patient's confidence in overcoming the disease, and cooperate with the treatment with a positive attitude. In terms of social support, actively communicate with patients' friends and colleagues, obtain their cooperation, and give patients comfort, encouragement, and support. Inform patients of possible advanced adverse reactions during radiotherapy and chemotherapy in advance, and pay attention to the care of adverse reactions [6]. First of all, it is necessary to closely monitor body temperature changes and duration, take body temperature every 4 hours, pay close attention to changes in the patient's mind, especially within 72 h after surgery, and pay attention to whether the patient has symptoms such as nausea, vomiting, and neck stiffness. The color and amount of the drainage fluid were observed, and the drainage tube was kept unobstructed. For patients with hyponatremia, closely monitor the changes in electrolytes after the operation to understand whether the patient has melena or vomiting blood, and pay attention to whether the complexion is pale and blood pressure drops, so as to detect the occurrence of gastrointestinal bleeding in time. If the patient has an adverse reaction, the nursing staff should follow the doctor's advice to give antiemetic, fluid replacement, and electrolyte treatments. Formulate a reasonable diet plan to ensure a normal supply of nutrients and improve the body's immunity. At the same time, strengthen functional exercises, enhance physical fitness, and improve the quality of life of patients. Both groups of patients were intervened until the patients were discharged.

### 2.4. Evaluation Index

#### 2.4.1. Nursing Satisfaction Score

After the two groups of nursing intervention, the hospital's self-made nursing satisfaction scale was used to evaluate the patient's nursing satisfaction, including two dimensions of nursing attitude and nursing skills. There are a total of 20 entries, each with a score of 1 to 5, with a full score of 100. The higher the score, the higher the nursing satisfaction. Scoring index: ≥85 is very satisfied, 60–85 is basically satisfied, and <60 is not satisfied.

#### 2.4.2. Quality of Life Score

Before and after the two groups of nursing intervention, the cancer quality of life core scale [7] was used to evaluate the quality of life of patients, including five areas of physiological function, social function, role function, cognitive function, and emotional function. The full score for each indicator is 100 points, and the total score is 500 points. The higher the score, the higher the quality of life.

#### 2.4.3. Sleep Quality

Before and after nursing intervention in the two groups, the time to fall asleep, sleep time, and the number of awakenings were recorded and compared. The shorter the time to fall asleep, the fewer the number of awakenings. The longer the patients sleep, the better the quality of sleep.

#### 2.4.4. Pain Degree Score

The morning after admission is recorded as T0, the morning one day before surgery (T1), the first day after surgery (T2), the seventh day after surgery (T3), and the morning before discharge (T4). The changes in body pain degree at different time points were compared between the two groups, and the visual simulation [8] (VAS) score was used. There are a total of 0–10 points, 0 is painless, and 10 is severe pain. The higher the score, the more severe the pain.

#### 2.4.5. Stress Indicator Level

Comparison of changes in body stress indicators at different time points: venous blood was drawn from patients for centrifugation, and radioimmunoassay was used to determine plasma cortisol (Cor) and adrenocorticotrophic hormone (ACTH) concentrations. The plasma C-reactive protein (CRP) concentration was determined by enzyme-linked immunosorbent assay (ELISA), and all steps were performed in accordance with the instructions.

#### 2.4.6. Bad Mood Score

Before and after the nursing intervention, the two groups were scored using the self-rating anxiety scale (SAS) and the self-rating depression scale (SDS) [9]. According to SAS and SDS, the anxiety and depression of the two groups of patients before and after nursing were evaluated. There are 20 items in SAS and SDS, and each item corresponds to 0 to 4 points. The higher the score, the more serious the anxiety and depression.

#### 2.4.7. Adverse Reactions

After nursing, observe and record the adverse reactions of the two groups of patients, including gastrointestinal reactions, bone marrow suppression, leukopenia, thrombocytopenia, and dizziness and nausea.

### 2.5. Statistical Methods

SPSS 23.0 statistical software was used to process the data. Technical data is expressed as *n* or %, and the *X*^2^ test is used for comparison between groups. Measurement data are expressed as mean ± standard deviation (SD), and *t*-test is used for comparison within and between groups. *P* < 0.05 is considered statistically significant.

## 3. Results

### 3.1. Comparison of Nursing Satisfaction between the Two Groups

After nursing, the nursing satisfaction degree of the control group was 80.85%, and the nursing satisfaction degree of the research group was 95.74%. The difference between the two groups was statistically significant (*X*^2^ = 11.678, *P*=0.003) (Table 2).

### 3.2. Comparison of Pain Degree and Sleep Quality between the Two Groups

There was no significant difference in VAS scores between the two groups of patients at T0 (*P* > 0.05). VAS scores increased at T1 and T2, while the VAS scores decreased at T3 and T4. And at T4, the VAS score of the research group decreased more significantly than that of the control group (*P* < 0.05). Before nursing, there was no significant difference in the time to fall asleep, sleep time, and number of awakenings between the two groups (*P* > 0.05). After nursing, the time to fall asleep and the number of awakenings of the two groups of patients showed an upward trend, and the increase in the control group was higher (*P* < 0.05). The sleep time of the two groups showed a downward trend, and the degree of decline of the control group was higher (*P* < 0.05), as shown in Figure 1 and Table 3.

Note: *t*_1_ and *P*_1_ indicate the comparison between the control group and before care, *t*_2_ and *P*_2_ indicate the comparison between the research group and before care, and *t*_3_ and *P*_3_ indicate the comparison between the two groups after care.

### 3.3. Comparison of Negative Emotions between the Two Groups before and after Nursing

Before nursing, there was no significant difference in SAS score and SDS score between the two groups (*P* > 0.05). After nursing, the SAS score and SDS score of the two groups decreased (^*∗*^*P* < 0.05), and the decrease in the research group was more obvious (^#^*P* < 0.05) (Figure 2).

### 3.4. Comparison of the Levels of Stress Indicators Cor, ACTH, and CRP between the Two Groups

There was no statistically significant difference in the levels of stress indicators Cor, ACTH, and CRP between the two groups at T1 (*P* > 0.05). With the passage of time, the levels of Cor and ACTH of the two groups showed an upward trend. At T4, the levels of Cor and ACTH in the research group increased less than those in the control group, and the difference was statistically significant (^*∗*^*P* < 0.05). The CRP levels of the two groups showed an upward trend at T1 and T2 and showed a downward trend at T3 and T4. And at T4, the CRP level of the research group decreased more than that of the control group, and the difference was statistically significant (^*∗*^*P* < 0.05) (Figure 3).

### 3.5. Comparison of the Quality of Life between the Two Groups before and after Nursing

Before nursing, there was no statistically significant difference between the two groups in physical function, social function, role function, cognitive function, emotional function, and total score (*P* > 0.05). After nursing, the scores of the quality of life indicators and total scores of the two groups increased, and the scores of the research group increased more significantly (*P* < 0.005) (Table 4).

### 3.6. Comparison of Adverse Reactions between the Two Groups

In the control group, there were 5 cases of gastrointestinal reactions, 7 cases of bone marrow suppression, 6 cases of leukopenia, 6 cases of thrombocytopenia, and 10 cases of dizziness and nausea. In the research group, there were 1 case of gastrointestinal reaction, 2 cases of bone marrow suppression, 1 case of leukopenia, 1 case of thrombocytopenia, and 2 cases of dizziness and nausea. The difference between the two groups was statistically significant (*P* < 0.05) (Table 5).

## 4. Discussion

Glioma is the most common primary tumor in the skull. Most patients with glioma are in the advanced stage when they see a doctor, which has a greater impact on the brain tissue of the patient and induces many complications. Glioma has a high fatality rate, which seriously affects the life safety of patients [10]. Clinically, surgical treatment is mainly used to treat glioma, although it can save the lives of patients. However, glioma is prone to recurrence after surgery, often supplemented by radiotherapy and chemotherapy [11, 12]. Although concurrent radiotherapy and chemotherapy can effectively kill tumor cells, the treatment will also bring different degrees of adverse reactions to the patients and aggravate the patients' anxiety, depression, and other unhealthy emotions, and the prognosis effect is not good. Coupled with the specificity of the location and treatment of glioma, it brings heavy pressure to the patient's body and psychology. Therefore, in addition to active treatment, the intervention of scientific and reasonable nursing mode is also very important for the negative emotions and common adverse reactions of patients with glioma during concurrent radiotherapy and chemotherapy [13]. According to the patient's condition and psychological characteristics, this research provides high-quality health education and psychological counseling. This study described in detail the relevant knowledge and precautions of glioma, which improved patients' awareness of their own disease and compliance with treatment, so that they could better cooperate with treatment and build confidence in overcoming the disease.

Studies have shown [14–16] that taking different psychological interventions before surgery to strengthen the cognitive function of patients has a significant effect on eliminating bad emotions. Studies have also shown [17, 18] that an effective care model can significantly reduce the incidence of adverse reactions in cancer chemotherapy patients and improve the tolerance and treatment confidence of patients with adverse reactions to chemotherapy. In this study, compared with the control group, the SAS and SDS scores of patients in the research group were significantly reduced after nursing. The VAS score increased significantly one day after surgery and decreased significantly when discharged from the hospital, and the research group was lower than the control group. After nursing, the scores of all dimensions of the quality of life and the total score were significantly improved, and the incidence of adverse reactions such as gastrointestinal reactions, leukopenia, and bone marrow suppression was significantly reduced, and the differences were statistically significant (*P* < 0.05). The results show that high-quality nursing intervention can significantly regulate the negative emotions of patients with glioma during concurrent radiotherapy and chemotherapy, reduce the degree of pain and the incidence of toxic side effects during concurrent radiotherapy and chemotherapy, effectively help patients to recover, and help improve the patient's physical and psychological conditions, and improve the patient's quality of life. In addition to providing professional psychological counseling and adverse reaction preventive care, nursing staff also need to earnestly implement the patient-centered nursing concept and improve the professional quality and nursing service capabilities of nursing staff, so as to provide patients with efficient and safe nursing services [19]. In this study, compared with the control group, patients in the research group were significantly more satisfied with nursing services than the control group (*P* < 0.05). The results show that high-quality nursing intervention can significantly improve the satisfaction of patients with glioma during concurrent radiotherapy and chemotherapy and improve the compliance of patients with treatment, which is conducive to the establishment of a good doctor-patient relationship and promotes the postoperative recovery of patients.

Both surgical stress and radiotherapy and chemotherapy stress can cause the patient's stress response, causing physiological and psychological abnormalities in the patient, resulting in neurological disorders; the adrenal medulla secretes catecholamines and abnormal sympathetic activity, which in turn leads to endocrine and immune system disorders [20, 21]. The body's stress response is physiologically mainly through the activation of the hypothalamus-pituitary-adrenal cortex endocrine axis and the sympathetic-adrenal medulla endocrine axis. Cor and ACTH are relatively sensitive indicators of the stress response, and detecting the levels of these two indicators in peripheral blood can reflect the patient's stress level [22, 23]. The concentration changes of the cytokine CRP are not only related to the direct stimulation of stress factors but also closely related to the neuroendocrine system [24, 25]. The results of this study showed that there was no statistically significant difference in the levels of stress indicators Cor, ACTH, and CRP between the two groups at T1. With the passage of time, the levels of Cor and ACTH of the two groups showed an upward trend. At T4, the increase in Cor and ACTH levels in the research group was less than those in the control group, and the difference was statistically significant. The CRP levels of the two groups showed an upward trend at T1 and T2 and showed a downward trend at T3 and T4. And at T4, the decrease in CRP level of the research group was greater than that of the control group, and the difference was statistically significant. The results suggest that patients with glioma have a stress response during surgery and concurrent radiotherapy and chemotherapy. The high-quality nursing measures used in this study can regulate the secretion of Cor, ACTH, and CRP, thereby inhibiting the degree of the stress response.

In short, high-quality nursing intervention can significantly alleviate the bad mood of patients with glioma during concurrent radiotherapy and chemotherapy and help improve the patient's stress response. High-quality nursing intervention can reduce the incidence of adverse reactions and pain levels, improve the quality of sleep and quality of life of patients, and increase the satisfaction with nursing services, which is worthy of clinical promotion. However, this study needs more research to confirm our conclusion, which is the limitation of this study.

## Figures and Tables

**Figure 1:** Comparison of VAS scores between the two groups. T0 means the morning after admission, T1 means the day before surgery, T2 means the first day after surgery, T3 means the seventh day after surgery, and T4 means the morning before discharge.

**Figure 2:** Comparison of the two groups of negative emotions. ^*∗*^*P* < 0.05 compared with before treatment; ^#^*P* < 0.05 compared with the control group. (a) The comparison of the two groups of SAS scores, and (b) the comparison of the two groups' SDS scores.

**Figure 3:** Comparison of the levels of stress indicators Cor, ACTH, and CRP between the two groups. ^*∗*^Compared with the control group, *P* < 0.05. (a) Comparison of Cor levels between the two groups, (b) comparison of ACTH levels between the two groups, and (c) comparison of CRP levels between the two groups.

**Table 1:** Comparison of general clinical data between the two groups.

Index	Control group (*n* = 47)	Research group (*n* = 47)	*X* ^2^	*P* value
Gender				
Male	29	26	0.394	>0.05
Female	18	21		

Age (year)				
>50	20	22	0.172	>0.05
≤50	27	25		

BMI (kg/m^2^)				
>22	29	31	0.184	>0.05
≤22	18	16		

Education level				
Senior high school and above	24	28	0.689	>0.05
Junior high school and below	23	19		

Tumor location				
Brain	32	34	0.294	>0.05
Cerebellum	5	5		
Diencephalon	4	3		
Cerebral ventricle	6	5		

**Table 2:** Comparison of nursing satisfaction between the two groups (*n*, %).

Groups	*n*	Very satisfied	Basic satisfaction	Dissatisfied	Satisfaction
Control group	47	12	26	9	38 (80.85)
Research group	47	27	18	2	45 (95.74)
*X* ^2^					11.678
*P* value					0.003

**Table 3:** Comparison of sleep quality between the two groups.

Groups		Time to fall asleep (min)	Sleeping time (h)	Number of awakenings (times)
Control group (*n* = 47)	Before nursing	45.37 ± 16.71	6.21 ± 1.42	2.36 ± 0.74
	After nursing	62.98 ± 18.36	4.16 ± 1.08	3.84 ± 0.82

Research group (*n* = 47)	Before nursing	46.15 ± 16.34	6.17 ± 1.47	2.41 ± 0.72
	After nursing	53.61 ± 17.48	5.25 ± 1.13	2.86 ± 0.77

*t*_1_		11.236	9.471	12.513
*P*_1_		≤0.001	0.001	0.002
*t*_2_		7.962	6.037	4.265
*P*_2_		0.002	0.012	0.036
*t*_3_		7.580	7.564	5.172
*P*_3_		0.001	0.007	0.014

**Table 4:** Comparison of quality of life between the two groups before and after nursing.

Index	Control group (*n* = 127)	Research group (*n* = 127)	t	*P* value
Physical function				
Before nursing	63.64 ± 5.23	62.71 ± 5.62	1.023	>0.05
After nursing	74.56 ± 6.36	89.36 ± 6.87	9.714	<0.05

Social function				
Before nursing	65.83 ± 5.24	66.29 ± 5.48	2.368	>0.05
After nursing	76.78 ± 7.62	91.32 ± 5.51	11.315	<0.05

Role function				
Before nursing	62.45 ± 5.68	62.91 ± 5.72	0.472	>0.05
After nursing	77.26 ± 6.82	87.23 ± 7.24	7.684	<0.05

Cognitive function				
Before nursing	66.35 ± 6.27	67.12 ± 6.54	0.937	>0.05
After nursing	78.36 ± 6.46	88.61 ± 6.58	5.238	<0.05

Emotional function				
Before nursing	60.73 ± 5.41	61.02 ± 5.65	0.670	>0.05
After nursing	73.26 ± 6.74	86.39 ± 6.88	6.663	<0.05

Total score				
Before nursing	323.58 ± 11.67	325.42 ± 10.73	1.392	>0.05
After nursing	391.62 ± 10.84	453.68 ± 12.83	14.273	<0.05

**Table 5:** Comparison of adverse reactions between the two groups.

Group	*n*	Gastrointestinal reaction	Bone marrow suppression	Leukopenia	Thrombocytopenia	Dizziness and nausea
Control group	47	5	7	6	6	10
Research group	47	1	2	1	1	2

## Data Availability

Data used to support the findings of this study are available on reasonable request to the corresponding author.
